This article has been retracted.

# POU Class 2 Associating Factor 1 Exerts a Protective Effect on the Respiratory Syncytial Virus-Induced Acute Bronchiolitis by the NF-*κ*B Pathway

**DOI:** 10.1155/2023/2815219

**Published:** 2023-05-23

**Authors:** Liwen Zhang, Zhiying Huang, Fei Wang, Mei Xue, Xiaoyu Zhang, Yu Wan, Liang Ma

**Affiliations:** ^1^Department of Pediatrics, The Second People's Hospital of Changzhou, Affiliated Hospital of Nanjing Medical University, Changzhou, Jiangsu, China; ^2^Department of Gastroenterology, The First People's Hospital of Changzhou, The Third Affiliated Hospital of Soochow University, Changzhou, Jiangsu, China

## Abstract

**Background:**

Respiratory syncytial virus (RSV) is the main pathogen causing acute bronchiolitis, which is common in infants and young children. A previous study revealed the possible involvement of POU class 2 associating factor 1 (POU2AF1) in RSV-triggered acute bronchiolitis. We attempted to clarify the specific action mechanism of POU2AF1 underlying RSV-triggered inflammation.

**Methods:**

RT-qPCR measured POU2AF1 levels in RSV-infected children, mice, and airway epithelial cell lines (HBECs). HE staining showed histopathological features in the lung tissue of RSV-infected mice. ELISA examined the contents of proinflammatory cytokines in RSV-infected mice. Western blotting evaluated the protein abundance of proinflammatory cytokines in RSV-infected HBECs and assessed NF-*κ*B pathway-associated protein expression in RSV-infected mice and RSV-treated HBECs.

**Results:**

POU2AF1 presented depletion in RSV-infected children, mice, and HBECs. RSV-infected triggered lung injury and inflammatory cell infiltration in the mouse lung tissue, while POU2AF1 overexpression rescued these changes. RSV-infected induced inflammatory impairment in HBECs, whereas POU2AF1 reversed this effect. POU2AF1 suppressed the upregulated NF-*κ*B pathway-associated protein expression in mice and HBECs under RSV infection.

**Conclusion:**

POU2AF1 exerts a protective impact on RSV-induced acute bronchiolitis in vitro and in vivo through the NF-*κ*B pathway. Our research may provide a novel direction for better therapy of RSV-triggered acute bronchiolitis.

## 1. Introduction

Acute bronchiolitis (bronchiolitis) is an acute lower respiratory tract infection common in infants and young children [1, 2], characterized by dyspnea, shortness of breath, and tissue hypoxia due to obstruction of the small airway [3]. According to multiple epidemiological investigations, respiratory syncytial virus (RSV) is the main pathogen causing bronchiolitis, with a high incidence in children under 6 months [4, 5]. Most bronchiolitis cases caused by RSV infection (RSV-induced bronchiolitis) occur in 2–5 months [6, 7]. So far, there are still no specific therapeutic strategies for bronchiolitis. After the lung tissue is infected by RSV, the exudation of tissue fluid caused by the inflammatory response causes lung edema and increases the lung mass [8]. Tissue fluid exudation secretes proinflammatory cytokines and releases inflammatory mediators such as TNF-*α*, IL-1*β*, etc., triggering an inflammatory cascade, and its activity reflects the pulmonary inflammatory response and the degree of damage [9]. Also, in bronchiolitis, proinflammatory cytokines TNF-*α*, IL-1*β*, IFN-*γ,* and IL-6 levels were found to be significantly enhanced [10, 11]. Thus, clarifying the molecular mechanism underlying the inflammatory response in the lung tissue after RSV infection is of significance for the therapy of bronchiolitis.

Up to date, ribavirin atomization, bronchodilators, etc., have all been applied to the therapy of bronchiolitis, but efficacy is quite controversial [12, 13]. Intravenous immunoglobulin and palivizumab are available for bronchiolitis prophylaxis. However, existing therapeutic drugs are expensive and limited to high-risk diseased children [14–16]. Therefore, the need for more reliable, cost-effective, and effective treatment is urgent. During the search for novel modulators of lung host defense by analyzing genome-wide RNA-seq data from normal human airway epithelium, POU domain class 2-associated factor 1 (POU2AF1), a known transcriptional cofactor, was previously thought to be expressed only in lymphocytes [17]. A study revealed a novel function of POU2AF1 as a potential modulator of host defense genes in human airway epithelium [18]. Previously, POU2AF1 was regarded as one of the predictive biomarkers of bronchiolitis obliterans syndrome over six months before diagnosis [19]. Moreover, POU2AF1 is downregulated in the blood of patients with end-stage chronic respiratory diseases [19]. Thus, we hypothesized that POU2AF1 may have a relationship with proinflammatory cytokines with a variety of biological functions in RSV-triggered bronchiolitis. In our previous research, we confirmed that suppression of the NF-*κ*B/IL-33/ST2 axis hindered the development of RSV-infected acute bronchiolitis [20]. Furthermore, when ST2 presents a combination with IL-33, it activates the NF-*κ*B pathway and facilitates the release of Th2 cytokines, including IL-4, IL-5, and IL-10 [21]. Thus, whether POU2AF1 modulates the NF-*κ*B pathway in RSV-triggered bronchiolitis needs further exploration.

Herein, we attempted to investigate POU2AF1's role underlying inflammation in RVS-triggered bronchiolitis and clarify its downstream pathway. We established animal models and cellular models to mimic characteristics of RVS-triggered bronchiolitis in vivo and in vitro. Our research may provide a novel insight for better therapy of RSV-triggered acute bronchiolitis.

## 2. Materials and Methods

### 2.1. Reagents, Antibodies, and Cell Lines

RSV from Hipower Pharmaceutical (Guangzhou, China); normal primary human bronchial epithelial cells (HBECs) collected from normal adults without diagnosed lung-related diseases with an approved protocol from Lifeline Cell Technology (Frederick, MD, USA); control cell line A549 from ATCC (USA); BALB/c mice from Guangdong Medical Animal Laboratory (Guangzhou, China); adenoviral (Adv) vectors from Hanbio (Shanghai, China); Lipofectamine 2000 from Invitrogen (USA); pcDNA POU2AF1 and pcDNA empty vectors from GenePharma (Shanghai, China); primary antibodies, including p-I*κ*Ba, p-p50, p-p65, I*κ*-Ba, p50, p65, TNF-*α*, IL-1*β*, IL-6, and GAPDH were purchased from Cell Signaling Technology (CA, USA); antirabbit horseradish peroxidase-labeled secondary antibodies from Abcam (Shanghai, China); RPMI1640 culture medium, fetal bovine serum (FBS), and 0.25% trypsin from Gibco (USA); penicillin and streptomycin from Thermo Fisher Scientific (USA); Trizol from Thermo Fisher Scientific (USA); Reverse transcriptase kit from Mingyang Kehua (Beijing, China); and SYBR PCR Master Mix kit from Shanghai Lianmai (Shanghai, China).

### 2.2. Study Subjects

Nasopharyngeal aspirates (NPAs) were collected from children hospitalized in the Second People's Hospital of Changzhou, Affiliated Hospital of Nanjing Medical University, due to acute respiratory symptoms such as coughing, wheezing, or tachypnea, from May 2019 to May 2021. Children with congenital heart disease, cardiopulmonary dysplasia, and immunodeficiency were excluded. Patients with other respiratory infections detected using a multiplex virus PCR panel or by serological testing were also excluded. A total of 22 children were finally enrolled in the study. There were 15 children who underwent physical examination in the same period who were recruited as the control group. There were no differences in age and gender between the control group and the RSV group. Respiratory symptoms were scored upon admission to assess the severity of respiratory illness. A sterile suction catheter was inserted into the oropharynx through the nostril using an electric suction pump for NPA collection. After washing the catheter with normal saline, specimens were stored in a viral transport medium at −70°C for use. The present study was approved by the ethics committee of the Second People's Hospital of Changzhou, Affiliated Hospital of Nanjing Medical University. All parents of subjects signed the written informed consent.

### 2.3. Animal Models

BALB/c mice (6–8 weeks old, 20 ± 1 g) were housed under specific pathogen-free conditions. They were randomly divided into 4 groups (*n* = 6 for each): the control group, the RSV group, the RSV + Adv-NC group, and the RSV + Adv-POU2AF1 group. The mice in the RSV infection group were anesthetized via intraperitoneal injection of 3% 0.1 ml/kg pentobarbital sodium, followed by a nasal drip of RSV with 100 ml of 10^6^ PFU for 6 consecutive days, whereas the mice in the control group were anesthetized via nasal drip of saline at the same dose. For delivery of the expressing Adv-POU2AF1 vector, mice in the RSV + Adv-NC and the RSV + Adv-POU2AF1 groups received intravenous injection of Adv-POU2AF1 (1 × 10^9^ PFU/100 *μ*L) or control Adv-NC (1 × 10^9^ PFU/100 *μ*L) once every 2 weeks for 6 weeks before RSV modeling. All the mice were sacrificed and whole-lung specimens were collected 3, 5, and 7 days after RSV infection. The animal study was approved by the animal care and use ethics committee of the Second People's Hospital of Changzhou, Affiliated Hospital of Nanjing Medical University.

### 2.4. Hematoxylin and Eosin (HE) Staining

Paraffin-embedded and sectioned mouse lung samples were stained with HE to assess inflammatory changes.

### 2.5. Enzyme Linked Immunosorbent Assay (ELISA)

The INF-*γ*, TNF-*α*, IL-1*β*, and IL-6 concentrations in mouse lung samples and cells were examined by corresponding ELISA kits (Cloud Clone Corp, Wuhan, China) under the manufacturer's guidance.

### 2.6. Cell Culture

HBECs and control cell line A549 were cultured in RPMI1640 medium containing 10% FBS, 100 U/ml penicillin, and 100 U/ml streptomycin at 37°C with 5% CO_2_, and cells at the logarithmic growth phase were taken for the following assays.

### 2.7. RNA Extraction and RT-qPCR

The total RNA was extracted from tissues and cells using TRIzol reagent. RNA concentration and purity were determined, followed by stem-loop reverse transcription. A reverse transcriptase kit was used for synthesizing cDNA, followed by PCR amplification. The SYBR PCR Master Mix kit was used for measuring gene expression. The primer sequences were listed as follows: POU2AF1 forward, 5′-GTGGTGCTGCCCCATCA-3′, and reverse 5′-GCAGACACAGAACCTTCCATGT-3′; IL-6 forward, 5′-ATGAACTCCTTCTCCACAAGCGC-3′, and reverse 5′-GAAGAGCCCTCAGGCTGGACTG-3′; GAPDH forward, 5′-ACCACAGTCCATGCCATCAC-3′, and reverse 5′-TCCACCACCCTGTTGCTGTA-3′. The relative expression of POU2AF1 and IL-6 were normalized to GAPDH using the 2^−ΔΔCT^ method.

### 2.8. Cell Transfection and RSV Stimulation

For RSV infection, cells were stimulated with RVS strain A2 (RSV-A2) at an MOI of 3 and incubated for 24 h. HBECs were transfected after 24 h of culture (37°C, 5% CO_2_). The cells were cultured to approximately 80% confluence in plates, and then transfected with POU2AF1 overexpression and empty vectors using Lipofectamine 2000 according to the manufacturer's instructions. After 48 h of transfection, the cells were harvested for the next assays.

### 2.9. Western Blot

The logarithmic phase HBECs were taken, the medium in the culture dish was aspirated, and the cells were stored in a sterile centrifuge tube. After centrifugation at 1200 r/min for 10 min, the lysate was added to resuspend the cells. The protein concentration was determined by the BCA method. The 5 × SDS gel electrophoresis buffer was added and denatured at 100°C for 10 min. After being completely separated by electrophoresis, the protein was transferred to the PVDF membrane by a semi-dry method. After blocking with 5% skimmed milk powder at room temperature for 2 h, the specific primary antibodies were added and incubated overnight at 4°C. Then the secondary antibodies were added, incubated for another 2 h, and washed with TBS. Absorbance analysis was performed after color development to calculate the relative expression of each protein.

### 2.10. Statistical Analysis

SPSS 20.0 software was used to process the data. The data were expressed as mean ± standard deviation. The mean of samples between two groups was compared using the *t*-test, and that of multiple groups using one-way analysis of variance followed by Tukey's posthoc test. Pearson correlation analysis assessed the relationship between POU2AF1 level and clinical symptom scores or between the POU2AF1 level and IL-6 level in NPA of RSV-infected children. The difference was statistically significant with *P* < 0.05.

## 3. Results

### 3.1. POU2AF1 Presents Downregulation in NPA of RSV-Infected Children

Previously, POU2AF1 was regarded as one of the predictive biomarkers of bronchiolitis obliterans syndrome over six months before diagnosis [19]. Thus, we wondered whether POU2AF1 exerted a role in underlying acute bronchiolitis after RSV infection. First, we enrolled 22 RSV-infected children and 15 controls according to inclusion and exclusion criteria (Figure 1(a)). NPA samples were collected from 22 RSV-infected children and 15 controls. Next, RT-qPCR measured POU2AF1 expression status in NPA of RSV-infected children. As a result, POU2AF1 exhibited depletion in NPA of RSV-infected children (Figure 1(b)). Additionally, RSV-infected children showed higher IL-6 levels in the RSV group relative to controls (Figure 1(c)), suggesting potential airway inflammation in RSV-infected children. The Pearson correlation analysis evaluated the association of POU2AF1 level and clinical symptom scores or IL-6 level. The results illustrated that the POU2AF1 level had a negative relationship to clinical symptom scores (Figure 1(d)) and IL-6 level in NPA of RSV-infected children (Figure 1(e)). Collectively, POU2AF1 presents depletion under RSV infection and has a relationship to the symptom severity of RSV-infected children. POU2AF1 may have an association with IL-6-triggered airway inflammation.

### 3.2. RSV Induces Lung Injury and Inflammation and Downregulates POU2AF1 in Mice

RSV-infected mouse models were constructed to mimic the characteristics of acute bronchiolitis in vivo. HE staining demonstrated the thick tracheal wall, wide intercellular space, and elevated perivascular and peribronchiolar inflammatory cell infiltration in mouse lung specimens (Figure 2(a)). Furthermore, neutrophil counts and monocyte counts presented elevation in mouse lung under RSV infection (Figure 2(b)-2(c)). Subsequently, ELISA measured the contents of proinflammatory cytokines in mouse lung tissue. The results depicted a marked elevation in INF-*γ*, TNF-*α*, IL-1*β,* and IL-6 concentrations in the mouse lung tissue under RSV infection (Figure 2(d)–2(g)). The above results indicated the successful construction of RSV mouse models. RT-qPCR illustrated the POU2AF1 depletion in the mouse lung tissue in RSV mice relative to controls (Figure 2(h)). Collectively, RSV facilitates lung injury, inflammatory cell recruitment, and proinflammatory cytokine production in mouse lung tissue.

### 3.3. POU2AF1 Attenuates Lung Injury and Inflammation in RSV-Infected Mice

Considering that inflammation was a vital consequence of RSV infection and POU2AF1 presented downregulation in the mouse lung tissue, we supposed that POU2AF1 might exert a protective role against inflammatory changes in RSV-infected mice. Thus, adv-POU2AF1 and adv-NC vectors were respectively injected into RSV-infected mice. RT-qPCR depicted the successful POU2AF1 knockdown in the lung tissue of RSV-infected mice (Figure 3(a)). Moreover, POU2AF1 attenuated lung injury and inflammatory cell infiltration (Figure 3(b)), rescued the elevated neutrophil and monocyte counts (Figure 3(c)-2(d)), and reversed the elevated INF-*γ*, TNF-*α*, IL-1*β,* and IL-6 concentrations in the lung tissue of RSV-infected mice (Figure 3(e)–3(h)). Collectively, POU2AF1 exerts a protective role against lung injury and inflammation in RSV-infected mice.

### 3.4. POU2AF1 Inactivates the NF-Κb Pathway in RSV-Infected Mice

In our previous research, NF-*κ*B/IL-33/ST2 axis mediates the RSV-infected acute bronchiolitis [20]. Thus, we wondered whether POU2AF1 exerts regulation in RSV-infected mice through the NF-*κ*B pathway. Western blotting demonstrated that RSV upregulated the phosphorylated I*κ*-Ba, p65, and p50 protein abundance in the mouse lung tissue, whereas POU2AF1 elevation countervailed such influence (Figure 4(a)–4(d)). Collectively, POU2AF1 suppresses NF-*κ*B pathway activation in RSV-infected mice.

### 3.5. POU2AF1 Ameliorates Inflammation in RSV-Infected Airway Epithelial Cells via the NF-Κb Pathway

RSV-infection cellular models were constructed in HBECs to mimic the characteristics of acute bronchiolitis in vitro. RT-qPCR illustrated that POU2AF1 presented downregulation under RSV treatment (Figure 5(a)). Additionally, the POU2AF1 level was elevated under transfection with pcDNA POU2AF1 plasmid (Figure 5(b)). Western blotting illustrated that TNF-*α*, IL-1*β,* and IL-6 protein abundance showed elevation under RSV stimulation and rescued by POU2AF1 overexpression (Figure 5(c)–5(e)). Furthermore, RSV facilitated I*κ*-Ba, p65, and p50 phosphorylation in the mouse lung tissue, whereas POU2AF1 upregulation counteracted such effect (Figures 5(f) and 5(g)). Collectively, POU2AF1 suppresses inflammation in vitro through the NF-*κ*B pathway.

## 4. Discussion

Respiratory viral infections, particularly RSV, are the most vital risk factor for wheezing onset among infants and young children [22]. Bronchiolitis is the most common acute respiratory infection in children younger than 1 year old and the most common reason for hospitalization in this age group [2, 22]. RSV accounts for approximately 70% of all bronchiolitis cases [23]. Herein, RSV infection induces airway inflammation in patients. RSV infection triggered lung impairment and inflammatory cell infiltration in vivo and facilitated inflammatory responses in vitro.

POU2AF1, a known B-cell transcriptional co-activator, exerts multiple roles in several diseases. For instance, POU2AF1 facilitates mesenchymal stem cell adipogenesis via HDAC1 downregulation [24]. POU2AF1 is involved in abdominal aortic aneurysm enlargement and has a predictive value for abdominal aortic aneurysm enlargement [25]. POU2AF1 presents elevation in B lymphocytes in idiopathic pulmonary fibrosis lungs and POU2AF1 deficiency protects mice from bleomycin-triggered lung fibrosis [17]. POU2AF1 is downregulated in the blood of patients with end-stage chronic respiratory diseases [19]. Herein, POU2AF1 presented downregulation in lung tissue from RSV-infected children and RSV-infected mice as well as RSV-treated airway epithelial cells, showing consistency with previous literature. Moreover, POU2AF1 overexpression rescued the airway inflammatory injury in RSV-infected mice. POU2AF1 elevation reversed the influence of RSV infection on airway epithelial cell inflammation. These findings suggest that POU2AF1 exerts a protective impact on RSV-triggered inflammatory injury in vitro and in vivo.

NF-*κ*B transcription factors are vital modulators of immunity, stress response, apoptosis, and differentiation [26]. Multiple stimuli combine with NF-*κ*B activation, which in turn mediates distinct transcriptional programs [26]. Thus, NF-*κ*B-dependent transcription signaling can be strictly controlled through positive and negative regulatory mechanisms. Previously, the NF-*κ*B pathway has been revealed to be involved in RSV-triggered inflammatory impairment. For instance, BRD4 couples NF-*κ*B/RelA with airway inflammatory response under RSV infection [27]. Another study revealed a great RSV-triggered p53/NF-*κ*B functional balance disequilibrium [28]. Herein, RSV infection facilitated expression elevation of NF-*κ*B pathway-related genes, p-I*κ*-Ba, p-65, and p50 in vitro and in vivo. POU2AF1 upregulation rescued these gene expression changes. These findings suggest that POU2AF1 facilitates RSV-triggered NF-*κ*B signaling inactivation in vitro and in vivo. However, the upstream mechanisms of POU2AF1 and other potential downstream pathways need further exploration in the future.

In conclusion, POU2AF1 ameliorates inflammation in RSV-infection-triggered acute bronchiolitis via the NF-*κ*B pathway, providing a potential novel insight for better therapy of RSV-triggered acute bronchiolitis.

## Figures and Tables

**Figure 1:** POU2AF1 presented downregulation in NPA of RSV-infected children. (a) Flow chart for grouping of RSV-infected children (*n* = 22) and controls (*n* = 15). (b) RT-qPCR detected POU2AF1 level in NPA of RSV-infected children and controls. (c) RT-qPCR detected IL-6 level in NPA of RSV-infected children and controls. (d) Pearson correlation analysis assessed relationship of POU2AF1 level and clinical symptom scores in NPA of RSV-infected children. (e) Pearson correlation analysis assessed relationship of POU2AF1 level and IL-6 level in NPA of RSV-infected children. ^*∗∗∗*^*P* < 0.001, RSV vs. Control group.

**Figure 2:** RSV-induced lung injury and inflammation and downregulated POU2AF1 in mice. (a) HE staining detected histopathological features in the lung tissue of RSV mice (*n* = 6) and controls (*n* = 6). (b, c) Cell counts for neutrophils and monocytes in the lung tissue of RSV mice and controls. (d–g) ELISA assessed INF-*γ*, TNF-*α*, IL-1*β,* and IL-6 concentrations in the lung tissue of RSV mice and controls. (h) RT-qPCR detected POU2AF1 level in RSV mice and controls. ^*∗∗∗*^*P* < 0.001, RSV vs. Control group.

**Figure 3:** POU2AF1 attenuated lung injury and inflammation in RSV-infected mice. (a) RT-qPCR measured POU2AF1 level in RSV mice after injection of adv-POU2AF1 (*n* = 6) and adv-NC (*n* = 6). (b) HE staining detected histopathological features in the lung tissue of RSV mice under POU2AF1 overexpression. (c, d) Cell counts for neutrophils and monocytes in the lung tissue of RSV mice under POU2AF1 overexpression. (e–h) ELISA assessed INF-*γ*, TNF-*α*, IL-1*β,* and IL-6 concentrations in the lung tissue of RSV mice under POU2AF1 overexpression. ^*∗∗*^*P* < 0.01, ^*∗∗∗*^*P* < 0.001, RSV + Adv-POU2FA1 vs. RSV + Adv-NC group.

**Figure 4:** POU2AF1 inactivated the NF-*κ*B pathway in RSV-infected mice. (a–d) Western blotting evaluated p-I*κ*-Ba, p-p65, p-p50, I*κ*-Ba, p65, and p50 protein abundance. ^*∗∗∗*^*P* < 0.001, RSV vs. Control group; ^###^*P* < 0.001, RSV + Adv-POU2FA1 vs. RSV + Adv-NC group.

**Figure 5:** POU2AF1 ameliorated inflammation in RSV-infected airway epithelial cells via the NF-*κ*B pathway. (a) RT-qPCR detected POU2AF1 level in RSV-treated HBECs and controls. (b) RT-qPCR detected POU2AF1 overexpression efficacy in RSV-treated HBECs. (c–e) Western blotting detected TNF-*α*, IL-1*β,* and IL-6 protein expressions under indicated treatment. (f, g) Western blotting detected p-I*κ*-Ba, p-p65, p-p50, I*κ*-Ba, p65, and p50 protein expressions under indicated treatment. ^*∗∗∗*^*P* < 0.001, RSV vs. Control group; ^###^*P* < 0.001, RSV + pcDNA POU2FA1 vs. RSV + pcDNA NC group.

## Data Availability

The data used to support the findings of this study are available from the corresponding author upon request.
